# The Relationship between Corporate Social Responsibility and Firm Value of Chinese Firms: Exploring from Degree of Internationalization

**DOI:** 10.1155/2023/7249799

**Published:** 2023-01-28

**Authors:** Renhong Wu, Md. Alamgir Hossain, Zhuoqi Teng, Xiangdong Shen

**Affiliations:** ^1^School of Management, Kyung Hee University, Seoul 02447, Republic of Korea; ^2^Department of Management, Hajee Mohammad Danesh Science and Technology University, Dinajpur 5200, Bangladesh; ^3^College of Business Administration, Henan Finance University, Zhengzhou 451464, China; ^4^Business School, Changshu Institute of Technology, Changshu 215500, China

## Abstract

The purpose of this paper is to explore the relationship between corporate social responsibility (CSR) and firm value in the Chinese market and identify factors that may influence it. We discuss the relationship between CSR engagement in Chinese firms and firm value from a nonlinear perspective. In addition, we examine how the degree of internationalization in a firm may affect the relationship between CSR and firm value. We employ the Hausman test to compare a random-effects and a fixed-effects model, and after testing and comparison, the fixed-effects model was chosen in our paper. Using data from 314 firms listed in China's A-shares market from 2010 to 2017, we verify the U-shaped relationship between CSR and firm value. Meanwhile, the degree of internationalization will affect firm value but cannot positively regulate the relationship between corporate social responsibility and firm value.

## 1. Introduction

Since the 1970s, the relationship between corporate social responsibility (CSR) and firm value has attracted the attention of scholars worldwide. Although research on the impact of CSR on firm value has been fruitful, there is still controversy regarding the results. The mainstream literature examines the relationship between CSR and firm value empirically using panel data. Most studies assume a linear or nonlinear relationship between these constructs and that a significant positive correlation exists between them [1]. In fact, most studies conclude that engagement in CSR activities is conducive to the improvement of firm value [2]. Waddock and Graves [3] put forward the concept of explicit and implicit costs, which demonstrates that firms that do not engage in CSR activities bear higher implicit and explicit costs and thus jeopardize their competitive advantage.

According to stakeholder theory, there is a two-way relationship between stakeholders and firms. The way to realize firm value is to prioritize the interests of stakeholders. Stakeholder pressure can prompt firms to take their social responsibilities seriously, which can significantly improve profitability and firm value [4, 5]. In practice, with the increasing concern about resources and the environment, human health, employee rights, and community development, engagement in CSR activities has become a universally accepted value in the business world.

Some believe that engagement in CSR activities is conducive to establishing a positive firm image, improving the firm reputation, and, in the long run, enhancing competitiveness, thus increasing firm value [6–8]. Ruf et al. [9], in an empirical study using the KLD database, find a positive correlation between engagement in CSR activities and firm value. Simpson and Kohers [10] identify a positive relationship between social performance and firm value in the context of US state-owned banks.

As for the motivations underlying the relationship between CSR and firm value, some scholars assert that engagement in CSR activities is not a simple form of altruism, but a win-win combination of altruism and egoism. Enterprises with a strong sense of social responsibility will actively introduce technology and increase their R&D investment to reduce resource consumption and costs, thereby improving firm value and working toward the corporate goal of maximizing profits while also preserving the environment. By contrast, if enterprises fail to pay attention to their social responsibilities or to maintain good relationships with various stakeholders, they may be unable to obtain resources and support and may suffer a loss of reputation, increased transaction costs, consumer resistance, brain drain, and various other problems, all of which reduce firm value.

Regarding the relationship between CSR and firm value, research conclusions to date mostly point to linear relationships. For example, Lu et al. [11] review studies conducted from 2002 to 2011, most of which identify a positive relationship between CSR and firm value. However, other researchers find a nonlinear relationship between CSR and firm value. For example, Wang et al. [12] studied 817 US companies listed in the Standard & Poor's Global Ratings and find a significantly inverted U-shaped relationship between engagement in CSR activities and firm value. However, Barnett and Salomon [13] find that there is a U-shaped relationship between CSR and firm value.

A literature review reveals that researchers have not yet reached a consensus on the relationship between CSR and firm value. Positive linear relationships, negative linear relationships, and curvilinear relationships have all been identified; curvilinear relationships have mostly been identified in the context of foreign-listed corporations. Western countries passed legislation on CSR fairly early, and their CSR systems are relatively complete. However, action in response to social responsibility in Chinese firms is still lacking. Research conclusions drawn by studying corporations operating in the West may not be applicable to the Chinese context.

Therefore, this study on the relationship between CSR and firm value seeks to address this research gap. Our paper makes three important contributions to the literature. First, from a localized perspective, we study the relationship between CSR and firm value in Chinese-listed enterprises to improve our understanding of the economic consequences of Chinese enterprises' engagement in CSR activities. Second, based on stakeholder theory and the microeconomic law of diminishing marginal returns, we explore the U-shaped relationship between engagement in CSR activities and firm value to deepen our understanding of this topic both in theory and in practice. Third, in the context of the international macroeconomic environment, we further examine the moderating role of the internationalization process in the relationship between CSR and firm value.

Based on the above-mentioned literature, this paper analyzes the value proposition of CSR engagement from the long-term perspective of sustainable competition based on stakeholder theory. The positive impacts of engagement in CSR activities may be unclear in the short term; meanwhile, such engagement may consume a certain amount of firms' wealth and resources and increase their operating costs. In the long run, however, such behavior will catch the attention of stakeholders and increase their trust, which not only enhances firms' reputation but also maintains good social relationships, thereby improving their future prospects. In addition, continuous engagement in CSR activities can enhance external and internal cohesion, which will eventually increase firm value.

After multinational enterprises enter the overseas market, their social identity changes and they inevitably face new problems. Fully understanding the rules, norms, and beliefs of the local market enables them to respond to the demands of stakeholders in the international market and be actively involved in CSR activities. In doing so, they overcome the liability of newness [14, 15], which in turn has a positive impact on firm value.

Considering CSR evaluation standards, a large number of studies use the quality of disclosed CSR reports to measure CSR performance. In this paper, we use the scores of a third-party ratings agency to measure CSR performance. This indicator not only allows us to analyze and evaluate the quality of information disclosed in the report but also includes specific content evaluation descriptors related to actual CSR performance activities.

Our paper is organized as follows.  Section 2 introduces the literature review and proposes our hypotheses.  Section 3 outlines the data collection method and explains the screening process.  Section 4 presents the results of our empirical study and tests the stability of the model through various methods.  Section 5 summarizes the conclusions based on the findings of the empirical analysis.

## 2. Theoretical Background and Research Hypotheses

### 2.1. CSR and Firm Value

Carroll [16] put forward four concepts related to CSR: economic responsibility, legal responsibility, ethical responsibility, and charitable responsibility and define them as follows: economic responsibility is the core responsibility of any business, legal responsibility implies that the firm must achieve economic goals within the limits of the law, ethical responsibility refers to the fact that firm behavior is consistent with social and ethical norms, and charitable responsibility is the CSR activities in which firms voluntarily engage. CSR may be narrowly defined as organizational responsibility to stakeholders other than shareholders. In a broad sense, CSR may be defined as the responsibility that all clearly defined stakeholders (including shareholders) associated with an organization should bear. CSR has always been a hot issue in academic research, not only in the economics and management fields but also in related fields. A large number of previous articles study CSR [13, 17–20], some of whom study the relationship between CSR and firm value [21–24].

According to stakeholder theory, meeting the needs of employees, customers, suppliers, organizations, and other groups is the key to rapid enterprise growth [25]. In addition, engagement in CSR activities as a typical stakeholder-oriented behavior can help enterprises establish and maintain good relationships with stakeholders and obtain more support and resources, which in turn gives them a competitive advantage and improves firm performance and value [26]. On one hand, from the perspective of consumers, firms that actively fulfill their social responsibilities are more likely to win the trust and goodwill of consumers, enhance consumers' willingness to purchase products, improve their reputation, and increase their market competitiveness. On the other hand, engaging in CSR activities can lead to being recognized by and receiving positive feedback from stakeholders such as shareholders, employees, customers, and suppliers, thereby maintaining a harmonious relationship with stakeholders, which also contributes to a sustainable competitive advantage [27]. It is also conducive to innovation and can be beneficial to human resources, firm reputation, organizational culture, and other intangible assets [28]. Finally, it can enable firms to achieve better performance and enhance their value.

Also, enterprises realize value creation through resource exchange with stakeholders. Thus, the better the relationship between a firm and its stakeholders, the more successful it will be. Engagement in CSR activities can improve the satisfaction of all stakeholders, thereby improving firm value [29]. For example, engagement in CSR activities can reduce businesses' risks and costs of capital; under these circumstances, suppliers are willing to provide higher-quality products and more preferential discounts. Enterprises with a sense of social responsibility are more likely to attract and motivate exceptional employees while reducing their labor costs [30], CSR can also improve consumer loyalty [31]. In addition, the government may put less pressure on enterprises that take their social responsibilities seriously [32]. When unexpected events occur, a good brand image can help weaken their negative influence. Active participation in CSR activities can bring about competitive advantages and encourage the formation of intangible assets such as innovation capabilities, human resources, reputation, and culture [28].

However, it is impossible to invest in CSR activities while also maintaining linear growth in terms of financial performance. According to the microeconomic rule of diminishing marginal returns, firms' growth in value diminishes as their investment in social responsibility increases [12]. While risk-averse corporate managers are prone to overinvest in CSR activities to reduce nonsystematic risks, shareholders can avoid such risks by diversifying their investment portfolios. Therefore, shareholders are often in favor of reducing involvement in CSR activities to make more risky investments that may increase firm value. Conversely, increasing investment in CSR activities at the expense of firm value may be the result of managers' personal motivations. When enterprises increase their investment in socially responsible activities, part of this expenditure is inevitably transferred to stakeholders, which leads to an increase in product prices and thus reduces investment returns. Although stakeholders with a sense of social responsibility may be willing to sacrifice a portion of their wealth to support socially responsible activities, they still expect reasonable returns. If their costs continue to increase and their financial returns continue to decrease, some stakeholders may begin to withdraw resources. That is, within a certain range of CSR investment, firm value increases, but once such investment exceeds a certain threshold, it tends to decrease. We, therefore, hypothesize the following.

  H1: There is an inverted U-shaped relationship between corporate social responsibility and firm value.

### 2.2. CSR and Firm Value of International Enterprises

Studies have shown that the internationalization of multinational Chinese enterprises is motivated by the desire to avoid domestic restrictions, seek new technologies and resource pools in the international market, realize value appreciation, and keep pace with competitors [33].

Multinational enterprises from developed countries are mainly responsible for the development of global social responsibility [34]. Such companies usually have a good image in their own countries and often choose CSR strategies based on the host country's emphasis on environmental protection or labor rights to strike a balance between the local and global responses. While international diversification makes multinational enterprises “better,” it also makes them “worse” [35]. Attig et al. [36] study 3,040 American companies and find a positive relationship between internationalization and CSR. The more the laws and regulations of the host country emphasizes social issues, the more obvious the role of internationalization in promoting CSR activities will be. In a study of British enterprises, Brammer et al. [37] reveal that the relationship between internationalization and CSR is not clear. Only when the host country has high CSR standards can internationalization increase engagement in socially responsible activities among multinational enterprises. Surroca et al. [38] note that the higher the expectations of stakeholders in the home country in terms of CSR, the greater the possibility that multinational enterprises will transfer their irresponsible practices to their subsidiaries.

The greater the degree of internationalization of multinational enterprises, the higher their commitment to overseas assets will be. This embeddedness in the overseas environment attracts attention and doubt from global stakeholders, which encourages enterprises to further increase their engagement in CSR activities to meet the demands of various stakeholders [36]. Not surprisingly, cultural and systemic differences shift their focus to social issues. The degree of internationalization affects the standards and expectations that multinational enterprises face. The greater the degree of internationalization, the more the expectations and demands of customers, investors, creditors, employees, regulatory agencies, and other stakeholders from the host country must be considered, and the broader the scope of CSR activities will be [39]. In addition, reputation has a contagious effect; for example, irresponsible behavior may initiate a chain reaction once it is discovered and made well known. Therefore, firms with a high degree of internationalization risk negative spillover from reputational damage [40].

For example, 19 US-listed Chinese enterprises were suspended or delisted in 2010 due to suspected financial fraud, which led to a crisis of trust in Chinese enterprises. In 2016, Alibaba's platform sales were delisted by the IACC, and the firm faced unprecedented public pressure and reputational loss in the international capital market. Zyglidopoulos et al. [41] demonstrate that the business activities of a multinational enterprise in one country affect its reputation and image in other countries and that actively fulfilling social responsibilities can alleviate those negative reputational impacts. Wang and Li [42] also point out that the reputations of multinational enterprises are no longer subject to geographical restrictions. Reputational damage may lead to the collapse of stakeholder trust and thus have a negative effect on firms' future business activities.

The problem of insufficient legal recognition has continued to affect multinational enterprises, which must constantly assert their commitment to legality to avoid adverse consequences and win greater support from stakeholders. Marano et al. [43] point out that undertaking CSR activities has become a mainstream business practice in the international market. In this study, we posit that the higher the degree of internationalization, the more firms will incorporate CSR activities into their regular operations. We, therefore, assert our formal hypothesis as follows.

  H2: The degree of internationalization positively affects the relationship between CSR and firm value.

## 3. Data, Variables, and Methodology

### 3.1. Sample and Data

For our sample, data for 314 firms listed on China's A-share market were collected for the 2010 to 2017 period. The data were drawn from two databases: Hexun.com's CSR and CSMAR (China Stock Market and Accounting Research) databases. Hexun.com is a representative third-party rating agency that measures CSR; it is similar to the KLD database but in the context of CSR. The CSMAR database organization is the first and largest professional high-tech firm engaged in the design and development of accurate financial and economic databases and has wide coverage, complete-time intervals, and rich indicators and is therefore the most widely used database in the Chinese academic community.

The selection process of the sample data in our paper is as follows. (1) Financial firms are excluded due to their unique characteristics; (2) ST (special treatment) and PT (particular transfer) firms are removed because they are financially abnormal and thus not comparable with other firms; (3) Firms whose data lacks continuity and those with missing information are excluded due to data insufficiency and other issues related to the firms themselves. For example, we were unable to collect rating data for many of the firms selected. Other data such as Tobin's *Q*, overseas sales revenue, total sales revenue, assets-to-liabilities ratio, firm ownership type, total assets, and other variables were obtained from the CSMAR database. Initially, data for more than 3,500 firms were obtained, but due to missing data in many cases, layer-by-layer screening was necessary. By matching data from the two databases by date and imposing multiple restriction conditions, we were able to obtain our sample data.

### 3.2. Research Model

#### 3.2.1. Dependent Variable

When resources are idle, firms are more likely to make charitable investments or engage in social activities. To account for stakeholders' power, we assert that the more engaged firms are in CSR activities, the more valuable they are. Because it offers many advantages, Tobin's *Q* is used to measure firm value in our paper. First, it is a prominent forward-looking indicator that reflects shareholders' expectations of a firm's future performance. Second, it is a combination of multiple firm performance variables, such as total sales, profits, cash flow, and net income. This comprehensive approach to firm performance provides reliable evidence of firm value. Third, it is an objective measure that does not reflect subjective evaluations of firm performance; therefore, it is the preferred indicator to measure the real value of a firm [44]. In this paper, Tobin's *Q* is calculated by taking the sum of the market value of equity and the book value of total liabilities, then dividing it by the book value of total assets. The result is used to measure the firm's economic performance and holdings of idle resources [45].

#### 3.2.2. Independent Variable

Multiple methods have been used to measure CSR, including several questionnaire methods [46]. Many scholars believe that self-disclosure largely reflects the extent of a firm's CSR activities, and most third parties (e.g., KLD, CASS, and SNAI) also consider the firm's self-reporting as important evidence of such activities [47]. This paper therefore also uses data from third-party rating agencies to measure CSR.

The dependent variable for this paper is the *t* + 1 period overall CSR score from Hexun.com. Scores range from 0 to 100; the higher the score, the higher the level of engagement in CSR activity. Hexun.com's CSR data have been used by many previous academic studies [22, 48]. Their Social Responsibility Index is a rating system divided into five first-level indicators: shareholder responsibility, customer and consumer rights responsibility, supplier and employee responsibility, environmental responsibility, and social responsibility. To ensure the scientific measurement of the CSR engagement of all A-share listed companies in the Shanghai and Shenzhen stock markets, second- and third-level indicators are included to complement first-level indicators. The second-level indicator contains 13 questions, and the third-level indicator contains 37 questions. This index has been recognized and used by many Chinese scholars for its accuracy and comprehensiveness.

#### 3.2.3. Moderator Variable

We use the ratio of overseas sales to total sales to measure of the degree of internationalization (DOI) of Chinese firms. On the one hand, it is a commonly used measure that directly reflects the extent of firms' internationalization and thus many western scholars have also adopted this indicator. On the other hand, due to data availability, most Chinese listed firms report overseas income and total income in their financial statements; thus, this ratio can be easily calculated. However, few firms disclose all information about their overseas subsidiaries. Although it is relatively easy to obtain DOI-related data, the acquisition of other data for international indicator data are more or less difficult. Like Attig et al. [36], Liu et al. [49] also use this calculation method to measure the DOI in their studies.

#### 3.2.4. Control Variable

We include several control variables because of their potential effect on the relationship between CSR and firm value. In previous studies [45], *Board Size* has been used as a control variable because it is related to firm value and CSR. Thus, it is used as a control variable in our paper. *Firm Size* is another control variable which has been shown to influence CSR and firm value [22, 24]. The reason for this is that large firms have a well-established reputation and attract stakeholder groups that demand more attention [50]. *Leverage* is also used as a control variable in our paper because the level of debt is related to both CSR and firm value [51]. For example, firms with higher debt levels may be more concerned with short-term goals such as profit maximization rather than long-term goals such as CSR [50]. Firms with a higher *R&D* intensity can achieve higher returns, and their unique technical knowledge and intangible assets may help them improve firm value [52]. Because the number of *Subsidiaries* with considerable operational autonomy may improve firm value [53], it is also included as a control variable in our paper.

### 3.3. Formatting of Mathematical Components

To test our hypotheses, panel data will be used to estimate the equations in this paper. The models for individual *I* = 1, 2, 3, 4,…, *N*, which is observed at times *t* = 1, 2, 3,…, *T*, are as follows:

(1) $$\begin{array}{c} {Tobin‘s\;Q}_{i,t+1}=\beta_{0}+\beta_{1}{BOARDSIZE}_{i,t}+\beta_{2}{FIRMSIZE}_{i,t}+\beta_{3}{LEV}_{i,t}+\beta_{4}{R\&D}_{i,t}+\beta_{5}{SUB}_{i,t}+\mu_{t}+\varepsilon_{i,t}\text{,} \end{array}$$

(2) $$\begin{array}{c} {Tobin‘s\;Q}_{i,t+1}=\beta_{0}+\beta_{1}{BOARDSIZE}_{i,t}+\beta_{2}{FIRMSIZE}_{i,t}+\beta_{3}{LEV}_{i,t}+\beta_{4}{R\&D}_{i,t}+\beta_{5}{SUB}_{i,t}+{\beta_{6}{CSR}_{i,t}+\mu }_{t}+\varepsilon_{i,t}\text{,} \end{array}$$

(3) $$\begin{array}{c} {Tobin‘s\;Q}_{i,t+1}=\beta_{0}+\beta_{1}{BOARDSIZE}_{i,t}+\beta_{2}{FIRMSIZE}_{i,t}+\beta_{3}{LEV}_{i,t}+\beta_{4}{R\&D}_{i,t}+\beta_{5}{SUB}_{i,t}+\beta_{6}{CSR}_{i,t}+\beta_{7}{{CSR}_{i,t}^{2}+\mu }_{t}+\varepsilon_{i,t}\text{,} \end{array}$$

(4) $$\begin{array}{c} {Tobin‘s\;Q}_{i,t+1}=\beta_{0}+\beta_{1}{BOARDSIZE}_{i,t}+\beta_{2}{FIRMSIZE}_{i,t}+\beta_{3}{LEV}_{i,t}+\beta_{4}{R\&D}_{i,t}+\beta_{5}{SUB}_{i,t}+\beta_{6}{CSR}_{i,t}+\beta_{7}{CSR}_{i,t}^{2}{+\beta_{8}{DOI}_{i,t}+\mu }_{t}+\varepsilon_{i,t}\text{.} \end{array}$$

In Models (1)–(4), Tobin's *Q*_*i,t+*1_ is the value of firm *i* at time *t + *1, CSR_*i,t*_ is the CSR score of firm *i* at time *t*, BOARDSIZE, FIRMSIZE, LEV, R&D, and SUB are control variables, DOI is the moderating variable, *μ*_*t*_ is the time-fixed effects, and *ε*_*i*,*t*_ is a random disturbance term.

## 4. Results

Table 1 presents the descriptive statistics for the dependent, independent, and control variables used in our study. It can be seen from the statistical results that the mean of Tobin's *Q* in our sample is 1.644 with a standard deviation of 1.481. The mean of CSR is 42.522, and its range is from 2.900 to 79.930, which shows that there is a large variance in the data for the observed firms. The mean of DOI is 0.212 with a standard deviation of 0.221, thus indicating that overseas sales are one of the most important sources of firms' operating income. The means of Board Size, Firm Size, Leverage, R&D, and Subsidiaries are 9.184, 0976, 0.491, 0.440, and 23.668, respectively.

Table 2 represents the Pearson correlation coefficient matrix of the main variables used in the model. The correlation coefficient between firm value (Tobin's *Q*) and CSR is −0.023, which is not significant; this implies that engagement in CSR activities can lower firm value, but this finding should be verified in another empirical model. The correlation coefficient between firm value (Tobin's *Q*) and DOI is 0.069, which differs from the findings of previous studies (e.g., −0.0106 and not significant in [54]; −0.14 in [55]), but it is within the 1% significance level. For greater accuracy and considering that it is a major issue in this paper, it will be tested in a subsequent model. As for the control variables, most of the correlation coefficients are significant and do not exceed 0.8, thus indicating that all meet the requirements of the model.

The multicollinearity problem cannot be ignored in an empirical regression analysis. If it is not controlled well, the accuracy of the results will be jeopardized. If the VIF values of the variables in the model exceed 10, it can be assumed that the model has multiple collinearity problems; if they are less than 10 but greater than one, it can be assumed that there is no multicollinearity problem. Moreover, TOL (tolerance) and VIF are closely linked, as TOL is the reciprocal of VIF. In the model, TOL ranges from zero to one; therefore, multicollinearity can also be measured using its values. If TOL is closer to zero, there is a much greater probability of multicollinearity. However, if TOL is closer to one, there is likely to be no multicollinearity problem. From Table 3, it can be seen that the maximum of VIF is 2.40, the mean is 1.410, and TOL ranges from 0.416 to 0.975. Consequently, we conclude that the multicollinearity problem does not exist in our empirical model.

Considering that we use panel data in our paper and to enhance the credibility of the results, we choose the hierarchical regression method in this paper. Also, we employ the Hausman test [56] to compare the random-effects and fixed-effects models (see Table 4 for the results), and after testing and comparison, the fixed-effects model was chosen in our paper. Meanwhile, the fixed-effects model can also partially control or solve the endogeneity problem to a certain extent [47].

Table 4 represents the regression results. Model 1 is a basic regression that includes all control variables. In Models 2 and 3, we add the main independent variable (CSR) to test H1. Model 4 is the full model, including all control and explanatory variables. In Model 2, the coefficient of CSR is −0.0067, and it is significant at the 1% level. This result indicates that in the pure linear relationship, engagement in CSR activities has a negative relationship with firm value (Tobin's *Q*). However, when we add the quadratic term of CSR in Model 3, its coefficient is −0.0247 (*p* < 0.01), the coefficient of CSR^2^ is 0.0002, and the significance level is 1%. This finding suggests that engagement in CSR activities can slow the growth of firm value (Tobin's *Q*) in the early stages, but this negative impact will become positive at a certain point. In other words, engagement in philanthropic activity requires firms to make economic sacrifices to a certain degree. Thus, in the early stages, as CSR activities increase, the firm value will decrease. Then, the firm value will increase once engagement in CSR activities exceeds a critical point because such engagement can benefit the firm by enhancing its brand image and reputation. Hence, engagement in CSR activities has a U-shaped rather than an inverted U-shaped relationship with firm value. Therefore, H1 is rejected. In Model 4, the coefficients of CSR and CSR^2^ are similar to those in Model 3 at the same significance levels, and the coefficient of DOI is −0.925 with a significance level of 5%. Thus, we conclude that as the DOI of Chinese firms improves, it negatively moderates the relationship between CSR and firm value. Therefore, H2 is rejected.

To ensure the robustness of the models and their results, we now run a series of robustness tests. First, according to the protocol followed by Ma et al. [47], we use the panel GLS method to rerun the regression. Because we utilize unbalanced panel data, the GLS method can accommodate heteroscedasticity and autocorrelation and avoid other interference factors. The results are reported in Table 5, where it can be seen that the U-shaped relationship between CSR and firm value (Tobin's *Q*) still exists and DOI negatively affects the relationship between CSR and firm value. Thus, the robustness tests indicate that the results have strong stability.

The Ohlson [57] model has often been used to test firm value [58–61], and it is useful to us because the firm value is our dependent variable. To check the robustness of DOI and firm value (H2), we extend and modify the basic Ohlson [57] model as follows:

(5) $$\begin{array}{c} {\;P}_{i,t+1}=\beta_{0}+\beta_{1}{EPS}_{i,t}+\beta_{2}{BPS}_{i,t}+\beta_{3}{BOARDSIZE}_{i,t}{+\beta }_{4}{FIRMSIZE}_{i,t}+\beta_{5}{LEV}_{i,t}+{\;\beta }_{6}{R\&D}_{i,t}+\beta_{7}{SUB}_{i,t}{+\beta_{8}{DOI}_{i,t}+\beta }_{9}{CSR}_{i,t}+\beta_{10}{CSR}_{i,t}^{2}{+\mu }_{t}+\varepsilon_{i,t}\text{,} \end{array}$$

where *P*_*i,t+*1_ is the end-of-day stock price three months after the end of the fiscal year, EPS_*i,t*_ is earnings per share of firm *i* at time *t*, BPS_i*,t*_ is book value per share of firm *i* at time *t*, BOARDSIZE_*i,t*_ is boardsize of firm *i* at time *t*, FIRMSIZE_*i,t*_ is the log total assets of firm *i* at time *t*, LEV_*i,t*_ is total debt/total assets of firm *i* at time *t*, R&D_*i,t*_ is the research and development expenses of firm *i* at time *t*, SUB_*i,t*_ is the number of subsidiaries a firm *i* at time *t*, DOI_*i,t*_ is the ratio of overseas sales to total sales a firm *i* at time *t*, CSR_*i,t*_ is the CSR score of firm *i* at time *t*, and *ε*_*i,t*_ is the error term.

The results are reported in Table 6. The values for EPS and BPS are significant at the 1% level in all models. The coefficients of *DOI* are −5.350, −5.022, and −4.955, respectively, and all values are statistically significant at the 5% level, which verifies our previous results. Furthermore, the U-shaped relationship between CSR and firm value is once again evident. Therefore, the verification methods used in our robustness tests further support the credibility of our empirical results.

## 5. Conclusions

Although the relationship between CSR and firm value has been widely studied, the results have been inconsistent. Most researchers follow instrumental stakeholder theory in analyzing the linear relationship between them. Both positive and negative relationships have been found in previous studies. We expand upon this research by focusing on nonlinear effects and using data from China, the largest developing country in the world. Sun et al. [23] identify an inverted U-shaped relationship between engagement in CSR activities and firm value by using American corporate data. The purposes of this paper are to explore the relationship between CSR and firm value in the context of the Chinese market and to identify other factors that may influence this relationship. We examine CSR engagement and firm value in Chinese firms from a nonlinear perspective, which is a novel approach. In addition, we include a moderating variable (DOI) in our empirical analysis as a factor that may affect the relationship between CSR and firm value. The contributions of this paper are as follows.

First, we find that there is a U-shaped relationship between CSR and firm value in China's listed companies, as opposed to Sun et al.'s [23] and Singh et al.'s [22] inverted U-shaped relationship. Engagement in CSR activities constitutes a social contribution that initially requires firms to sacrifice their economic benefits to some extent; for this reason, firm value declines with an increase in CSR activities in the early stages. On the one hand, although engagement in CSR activities may balance the interests of various stakeholders, these interests are not easily reconciled. When engagement in CSR activities exceeds a certain level, firms may benefit not only in terms of tangible assets but also in terms of intangible assets. On the other hand, related investments may improve production efficiency, thereby leading to a reputational upgrade. In the second stage, CSR improves firm value. Hence, the relationship between CSR and firm value is most accurately represented by a U-shaped curve. China is the largest emerging economy in the world, with a unique market environment and other factors that influence firm value, and Chinese firms have not encountered the same problems as American firms. As such, the results may be quite different from those in a Western context.

Second, although many factors affect the relationship between CSR and firm value, we study it from an international perspective by analyzing the degree of internationalization (DOI). Although some studies have been conducted on the influence of DOI on firm value [62, 63], some scholars have studied CSR from the perspective of DOI in recent years [36, 64]. Our research reveals that DOI undermines firm value because Chinese firms that have access to international markets encounter a series of obstacles such as the liability of foreignness, product popularity, and trade protection policies in the host country. Due to these obstacles, DOI will affect firm value but cannot positively regulate the relationship between CSR and firm value. Still, this finding contributes to the research on CSR and firm value.

This paper has both theoretical and managerial implications. Regarding its theoretical implications, our paper extends the application of stakeholder theory in the context of CSR. In previous research, stakeholder theory has been used to study CSR engagement [65]. Specifically, some stakeholders (such as consumers) may strongly penalize businesses in the short term, while other stakeholders, such as long-term investors, may not view engagement in CSR as a firm risk. Thus, stakeholder relationships are a resource advantage that can be used to create competitive advantages [26]. As this study is based on stakeholder theory, we consider the nature of the relationship between vertical stakeholders and firms rather than a simple set of short-term relationships. This paper studies Chinese listed firms from the perspective of stakeholder theory, which is a setting conducive to studying the relationship between CSR and firm value. Also, CSR engagement can promote sustainable development [66], which may improve firm value in the long term. Engagement in CSR activities, as an indispensable key to firm performance, clearly affects firm value. In our paper, the results do not generate the inverted U-shaped relationship as identified in [23]. However, our results lay a foundation for future researchers to follow in considering the relationship between CSR and firm value and how DOI affects that relationship.

Our results also indicate that business leaders and management practitioners should change their traditional ideas such that they have a sense of long-term development. Because there is a U-shaped relationship between CSR and firm value, if business managers focus only on their companies' short-term interests, the effect of engaging in CSR on firm value will be minimal and its positive effects will only be evident in the second stage; therefore, long-term management vision is necessary. Also, DOI is a reality that Chinese firms cannot avoid, although it will hinder the relationship between engagement in CSR and firm value to some extent in the short term. From a long-term strategic point of view, DOI will bring benefits to firms, such as broader market access and access to global resources. Accordingly, business managers should have the confidence and persistence to manage their firms not only to balance the interests of all stakeholders, but also to encourage employees to realize their value in the company and foster relationships among customers, employees, investors, and other stakeholders to achieve common goals. DOI also promotes the active pursuit of technological innovation while increasing R&D investment and long-term competitive advantages, all of which help to improve firm value.

Finally, despite our careful research design, rigorous empirical study, and important contributions, several limitations exist that point to the need for future research. First, our research sample consisted of listed firms from the country with the largest developing economy, that is, China. Because of China's special market conditions and economic environment, the results may not be representative of other emerging countries. Future studies should utilize samples from different emerging countries or developing countries to make a horizontal comparison and reach a universal conclusion. Second, our paper is limited by indicator selection. That is, CSR data are scored by the Hexun rating, and although this method has been widely used in previous studies, it may not be universal because we use only the total score. Also, our DOI variable is represented by the ratio of overseas sales revenue to total income; thus, it exhibits a certain degree of unilateralism. Hence, future studies should choose the date indicator from a more representative and diversified database and collect data through other channels such as a field or questionnaire surveys to obtain more complete data. Third, the sample firms used in our research include those involved in the stock market, but some corporations with international influence such as Huawei are not publicly listed. Future studies should be extended to include nonlisted firms, nonpublic firms, and even small and medium-sized enterprises with multinational operations. Although many nonlisted firms do not publish annual reports, data may be collected through questionnaires or field visits to ensure the credibility and practicality of the results. Fourth, our paper ignores a very important distinction between state-owned enterprises (SOEs) and nonstate-owned enterprises (non-SOEs). In future research, this distinction should be fully taken into consideration; data from firms in different industries such as the services, manufacturing, and petrochemical industries may also be considered, and specific research on transnational operations in different industries may be conducted.

## Figures and Tables

**Table 1:** Descriptive statistics.

Variable	Mean	Std. dev	Min	Max
Tobin's *Q*	1.644	1.481	0.000	8.073
Board size	9.184	1.811	5.000	15.000
Firm size	0.976	0.643	−0.187	2.741
Leverage	0.491	0.196	0.077	0.887
R&D	0.440	1.176	0.000	8.371
Subsidiaries	23.668	26.790	1.000	158.000
CSR	42.522	22.091	2.900	79.930
DOI	0.212	0.221	0.001	0.912

**Table 2:** Pearson correlation matrix.

Variables	Tobin's *Q*	Board Size	Firm Size	Leverage	R&D	Subsidiaries	CSR	DOI
Tobin's *Q*	1							
Board size	−0.115^*∗∗∗*^	1						
Firm size	−0.498^*∗∗∗*^	0.175^*∗∗∗*^	1					
Leverage	−0.562^*∗∗∗*^	0.099^*∗∗∗*^	0.546^*∗∗∗*^	1				
R&D	−0.200^*∗∗∗*^	0.005	0.554^*∗∗∗*^	0.266^*∗∗∗*^	1			
Subsidiaries	−0.204^*∗∗∗*^	−0.002	0.521^*∗∗∗*^	0.233^*∗∗∗*^	0.378^*∗∗∗*^	1		
CSR	−0.023	0.057^*∗∗∗*^	0.066^*∗∗∗*^	−0.056^*∗∗∗*^	−0.022	−0.058^*∗∗∗*^	1	
DOI	0.069^*∗∗∗*^	−0.027	−0.143^*∗∗∗*^	−0.074^*∗∗∗*^	−0.044^*∗∗*^	−0.077^*∗∗∗*^	0.010	1

^*∗∗∗*^ *p* < 0.01, ^*∗∗*^*p* < 0.05, ^*∗*^*p* < 0.1.

**Table 3:** Collinearity test results.

Variable	VIF	1/VIF
Firm size	2.400	0.416
R&D	1.490	0.672
Leverage	1.470	0.682
Subsidiaries	1.400	0.714
Board Size	1.060	0.947
CSR	1.040	0.963
DOI	1.030	0.975

**Table 4:** Regression results.

	(1)	(2)	(3)	(4)
Board size	−0.00768	−0.0018	0.000948	−0.00265
	[0.021]	[0.022]	[0.022]	[0.022]
Firm size	−0.899^*∗∗∗*^	−0.880^*∗∗∗*^	−0.900^*∗∗∗*^	−0.887^*∗∗∗*^
	[0.296]	[0.295]	[0.299]	[0.294]
Leverage	−0.382	−0.530^*∗*^	−0.597^*∗*^	−0.571^*∗*^
	[0.302]	[0.309]	[0.314]	[0.312]
R&D	0.025	−3.3*E* − 05	0.00231	0.00974
	[0.020]	[0.020]	[0.020]	[0.021]
Subsidiaries	0.00434^*∗∗∗*^	0.00349^*∗∗∗*^	0.00307^*∗∗*^	0.00307^*∗∗*^
	[0.001]	[0.001]	[0.001]	[0.001]
CSR		−0.00674^*∗∗∗*^	−0.0247^*∗∗∗*^	−0.0247^*∗∗∗*^
		[0.001]	[0.006]	[0.006]
CSR^2^			0.000208^*∗∗∗*^	0.000207^*∗∗∗*^
			[0.000]	[0.000]
DOI				−0.925^*∗∗*^
				[0.390]
Constant	2.610^*∗∗∗*^	2.944^*∗∗∗*^	3.265^*∗∗∗*^	3.463^*∗∗∗*^
	[0.373]	[0.409]	[0.460]	[0.473]
Hausman	52.720^*∗∗∗*^	55.330^*∗∗∗*^	53.030^*∗∗∗*^	60.700^*∗∗∗*^
*N*	2000	1947	1947	1947
Adj. *R*^2^	0.027	0.058	0.066	0.073
Year	Yes	Yes	Yes	Yes
Firms	Yes	Yes	Yes	Yes

Standard errors in brackets; ^*∗∗∗*^*p* < 0.01, ^*∗∗*^*p* < 0.05, ^*∗*^*p* < 0.1.

**Table 5:** Robustness check: GLS method.

	(1)	(2)	(3)	(4)
Board size	0.068	0.031	0.029	0.036
	[0.137]	[0.139]	[0.138]	[0.138]
Firm size	−2.792^*∗∗∗*^	−2.736^*∗∗∗*^	−2.857^*∗∗∗*^	−3.102^*∗∗∗*^
	[0.579]	[0.598]	[0.599]	[0.602]
Leverage	−10.700^*∗∗∗*^	−10.500^*∗∗∗*^	−10.450^*∗∗∗*^	−10.400^*∗∗∗*^
	[1.486]	[1.545]	[1.543]	[1.538]
R&D	0.567^*∗∗∗*^	0.497^*∗∗∗*^	0.529^*∗∗∗*^	0.570^*∗∗∗*^
	[0.256]	[0.262]	[0.011]	[0.261]
Subsidiaries	0.060^*∗∗∗*^	0.061^*∗∗∗*^	0.059^*∗∗∗*^	0.059^*∗∗∗*^
	[0.011]	[0.011]	[0.011]	[0.011]
CSR		−0.026^*∗∗∗*^	−0.130^*∗∗∗*^	−0.123^*∗∗∗*^
		[0.011]	[0.059]	[0.059]
CSR^2^			0.00182^*∗∗*^	0.00176^*∗∗*^
			[0.001]	[0.001]
DOI				−3.886^*∗∗∗*^
				[1.143]
Constant	20.120^*∗∗∗*^	19.150^*∗∗∗*^	21.700^*∗∗∗*^	22.500^*∗∗∗*^
	[1.375]	[1.485]	[1.762]	[1.773]
*N*	2000	1947	1947	1947

Standard errors in brackets; ^*∗∗∗*^*p* < 0.01, ^*∗∗*^*p* < 0.05, ^*∗*^*p* < 0.1.

**Table 6:** Robustness check: Ohlson model.

	(1)	(2)	(3)
EPS	2.437^*∗∗∗*^	3.185^*∗∗∗*^	3.187^*∗∗∗*^
	[0.517]	[0.624]	[0.619]
BPS	0.674^*∗∗∗*^	0.593^*∗∗∗*^	0.618^*∗∗∗*^
	[0.186]	[0.188]	[0.189]
Board size	−0.148	−0.106	−0.0879
	[0.186]	[0.194]	[0.194]
Firm size	−3.733^*∗∗*^	−3.407^*∗∗*^	−3.590^*∗∗*^
	[1.640]	[1.623]	[1.626]
Leverage	12.01^*∗∗∗*^	11.13^*∗∗∗*^	10.83^*∗∗∗*^
	[2.355]	[2.423]	[2.438]
R&D	0.224	0.0723	0.0836
	[0.231]	[0.231]	[0.230]
Subsidiaries	0.049^*∗∗∗*^	0.046^*∗∗∗*^	0.043^*∗∗∗*^
	[0.011]	[0.011]	[0.011]
DOI	−5.350^*∗∗*^	−5.022^*∗∗*^	−4.955^*∗∗*^
	[2.303]	[2.247]	[2.323]
CSR		−0.0358^*∗∗∗*^	−0.158^*∗∗∗*^
		[0.009]	[0.038]
CSR^2^			0.00142^*∗∗∗*^
			[0.000]
Constant	8.845^*∗∗∗*^	10.30^*∗∗∗*^	12.34^*∗∗∗*^
	[2.661]	[2.876]	[2.902]
*N*	2000	1947	1947
Adj. *R*^2^	0.096	0.114	0.119
Year	Yes	Yes	Yes
Firms	Yes	Yes	Yes

Standard errors in brackets; ^*∗∗∗*^*p* < 0.01, ^*∗∗*^*p* < 0.05, ^*∗*^*p* < 0.1.

## Data Availability

The data used to support the findings of this study are available from the corresponding author upon request.

## References

[1] Johnson H. H. (2003). Does it pay to be good? Social responsibility and financial performance. *Business Horizons*.

[2] Blacconiere W. G., Patten D. M. (1994). Environmental disclosures, regulatory costs, and changes in firm value. *Journal of Accounting and Economics*.

[3] Waddock S. A., Graves S. B. (1997). The corporate social performance–financial performance link. *Strategic Management Journal*.

[4] Bocquet R., Le Bas C., Mothe C., Poussing N. (2017). CSR, innovation, and firm performance in sluggish growth contexts: a firm-level empirical analysis. *Journal of Business Ethics*.

[5] Cook K. A., Romi A. M., Sánchez D., Sánchez J. M. (2019). The influence of corporate social responsibility on investment efficiency and innovation. *Journal of Business Finance & Accounting*.

[6] Mishra S., Suar D. (2010). Does corporate social responsibility influence firm performance of Indian companies?. *Journal of Business Ethics*.

[7] Sun W., Cui K. (2014). Linking corporate social responsibility to firm default risk. *European Management Journal*.

[8] Saeidi S. P., Sofian S., Saeidi P., Saeidi S. P., Saaeidi S. A. (2015). How does corporate social responsibility contribute to firm financial performance? The mediating role of competitive advantage, reputation, and customer satisfaction. *Journal of business research*.

[9] Ruf B. M., Muralidhar K., Brown R. M., Janney J. J., Paul K. (2001). An empirical investigation of the relationship between change in corporate social performance and financial performance: a stakeholder theory perspective. *Journal of Business Ethics*.

[10] Simpson W. G., Kohers T. (2002). The link between corporate social and financial performance: evidence from the banking industry. *Journal of Business Ethics*.

[11] Lu W., Chau K. W., Wang H., Pan W. (2014). A decade’s debate on the nexus between corporate social and corporate financial performance: a critical review of empirical studies 2002–2011. *Journal of Cleaner Production*.

[12] Wang H., Choi J., Li J. (2008). Too little or too much? untangling the relationship between corporate philanthropy and firm financial performance. *Organization Science*.

[13] Barnett M. L., Salomon R. M. (2012). Does it pay to be really good? addressing the shape of the relationship between social and financial performance. *Strategic Management Journal*.

[14] Pant A., Ramachandran J. (2012). Legitimacy beyond borders: I ndian software services firms in the United States, 1984 to 2004. *Global Strategy Journal*.

[15] Madhok A., Keyhani M. (2012). Acquisitions as entrepreneurship: asymmetries, opportunities, and the internationalization of multinationals from emerging economies. *Global Strategy Journal*.

[16] Carroll A. B. (1979). A three-dimensional conceptual model of corporate performance. *Academy of Management Review*.

[17] Ting I. W. K., Azizan N. A., Bhaskaran R. K., Sukumaran S. K. (2019). Corporate social performance and firm performance: comparative study among developed and emerging market firms. *Sustainability*.

[18] Chen C.-J., Guo R.-S., Hsiao Y.-C., Chen K.-L. (2018). How business strategy in non-financial firms moderates the curvilinear effects of corporate social responsibility and irresponsibility on corporate financial performance. *Journal of Business Research*.

[19] Lin W. L., Law S. H., Azman-Saini W. N. W. (2020). Market differentiation threshold and the relationship between corporate social responsibility and corporate financial performance. *Corporate Social Responsibility and Environmental Management*.

[20] Ali H. Y., Danish R. Q., Asrar-ul-Haq M. (2020). How corporate social responsibility boosts firm financial performance: the mediating role of corporate image and customer satisfaction. *Corporate Social Responsibility and Environmental Management*.

[21] Qureshi M. A., Kirkerud S., Theresa K., Ahsan T. (2019). The impact of sustainability (environmental, social, and governance) disclosure and board diversity on firm value: the moderating role of industry sensitivity. *Business Strategy and the Environment*.

[22] Singh P. J., Sethuraman K., Lam J. Y. (2017). Impact of corporate social responsibility dimensions on firm value: some evidence from Hong Kong and China. *Sustainability*.

[23] Sun W., Yao S., Govind R. (2019). Reexamining corporate social responsibility and shareholder value: the inverted-U-shaped relationship and the moderation of marketing capability. *Journal of Business Ethics*.

[24] D’Amato A., Falivena C. (2020). Corporate social responsibility and firm value: do firm size and age matter? Empirical evidence from European listed companies. *Corporate Social Responsibility and Environmental Management*.

[25] Donaldson T., Preston L. E. (1995). The stakeholder theory of the corporation: concepts, evidence, and implications. *Academy of Management Review*.

[26] Jones T. M. (1995). Instrumental stakeholder theory: a synthesis of ethics and economics. *Academy of Management Review*.

[27] Maignan I., Ferrell O. C. (2004). Corporate social responsibility and marketing: an integrative framework. *Journal of the Academy of Marketing Science*.

[28] Surroca J., Tribó J. A., Waddock S. (2010). Corporate responsibility and financial performance: the role of intangible resources. *Strategic Management Journal*.

[29] Aaver B., Cadez S., Cadez S. (2009). Management accountants’ participation in strategic management process: a cross – industry comparision. *Journal for East European Management Studies*.

[30] Albinger H. S., Freeman S. J. (2000). Corporate social performance and attractiveness as an employer to different job seeking populations. *Journal of Business Ethics*.

[31] Castaldo S., Perrini F., Misani N., Tencati A. (2009). The missing link between corporate social responsibility and consumer trust: the case of fair trade products. *Journal of Business Ethics*.

[32] Hillman A. J., Keim G. D. (2001). Shareholder value, stakeholder management, and social issues: what’s the bottom line?. *Strategic Management Journal*.

[33] Ramamurti R., Hillemann J. (2018). What is ‘Chinese’ about Chinese multinationals?. *Journal of International Business Studies*.

[34] Gugler P., Shi J. Y. J. (2009). Corporate social responsibility for developing country multinational corporations: lost war in pertaining global competitiveness?. *Journal of Business Ethics*.

[35] Strike V. M., Gao J., Bansal P. (2006). Being good while being bad: social responsibility and the international diversification of US firms. *Journal of International Business Studies*.

[36] Attig N., Boubakri N., El Ghoul S., Guedhami O. (2016). Firm internationalization and corporate social responsibility. *Journal of Business Ethics*.

[37] Brammer S. J., Pavelin S., Porter L. A. (2009). Corporate charitable giving, multinational companies and countries of concern. *Journal of Management Studies*.

[38] Surroca J., Tribó J. A., Zahra S. A. (2013). Stakeholder pressure on MNEs and the transfer of socially irresponsible practices to subsidiaries. *Academy of Management Journal*.

[39] Kang J. (2013). The relationship between corporate diversification and corporate social performance. *Strategic Management Journal*.

[40] Fiaschi D., Giuliani E., Nieri F. (2017). Overcoming the liability of origin by doing no-harm: emerging country firms’ social irresponsibility as they go global. *Journal of World Business*.

[41] Zyglidopoulos S., Williamson P., Symeou P. (2016). The corporate social performance of developing country multinationals. *Business Ethics Quarterly*.

[42] Wang S. L., Li D. (2019). Responding to public disclosure of corporate social irresponsibility in host countries: information control and ownership control. *Journal of International Business Studies*.

[43] Marano V., Tashman P., Kostova T. (2017). Escaping the iron cage: liabilities of origin and CSR reporting of emerging market multinational enterprises. *Journal of International Business Studies*.

[44] Price J. M., Sun W. (2017). Doing good and doing bad: the impact of corporate social responsibility and irresponsibility on firm performance. *Journal of Business Research*.

[45] Li D., Lin H., Yang Y. w. (2016). Does the stakeholders–corporate social responsibility (CSR) relationship exist in emerging countries? Evidence from China. *Social Responsibility Journal*.

[46] Bondy K., Starkey K. (2014). The dilemmas of internationalization: corporate social responsibility in the multinational corporation. *British Journal of Management*.

[47] Ma H., Zeng S., Shen G. Q., Lin H., Chen H. (2016). International diversification and corporate social responsibility: an empirical study of Chinese contractors. *Management Decision*.

[48] Shahab Y., Ntim C. G., Ullah F. (2019). The brighter side of being socially responsible: CSR ratings and financial distress among Chinese state and non-state owned firms. *Applied Economics Letters*.

[49] Liu H., Luo J. h., Cui V. (2018). The impact of internationalization on home country charitable donation: evidence from Chinese firms. *Management International Review*.

[50] Hu Y., Zhu Y., Hu Y. (2016). Does ownership type matter for corporate social responsibility disclosure: evidence from China. *Global Conference on Business and Finance Proceedings*.

[51] Mishra D. R. (2017). Post-innovation CSR performance and firm value. *Journal of Business Ethics*.

[52] Schnippering M. (2020). R&D: the missing link between corporate social performance and financial performance?. *Management Review Quarterly*.

[53] Ambos T. C., Birkinshaw J. (2010). Headquarters’ attention and its effect on subsidiary performance. *Management International Review*.

[54] Chen S., Tan H. (2012). Region effects in the internationalization–performance relationship in Chinese firms. *Journal of World Business*.

[55] Ma X., Yiu D. W., Zhou N. (2014). Facing global economic crisis: foreign sales, ownership groups, and corporate value. *Journal of World Business*.

[56] Hausman J. A. (1978). Specification tests in econometrics,” Econometrica. *Journal of the Econometric Society*.

[57] Ohlson J. A. (1995). Earnings, book values, and dividends in equity valuation. *Contemporary Accounting Research*.

[58] Grassmann M. (2021). The relationship between corporate social responsibility expenditures and firm value: the moderating role of integrated reporting. *Journal of Cleaner Production*.

[59] Sinkin C., Wright C. J., Burnett R. D. (2008). Eco-efficiency and firm value. *Journal of Accounting and Public Policy*.

[60] Schadewitz H., Niskala M. (2010). Communication via responsibility reporting and its effect on firm value in Finland. *Corporate Social Responsibility and Environmental Management*.

[61] Gregory A., Whittaker J., Yan X. (2016). Corporate social performance, competitive advantage, earnings persistence and firm value. *Journal of Business Finance & Accounting*.

[62] Mendoza X., Espinosa-Méndez C., Araya-Castillo L. (2020). When geography matters: international diversification and firm performance of Spanish multinationals. *BRQ Business Research Quarterly*.

[63] Pisani N., Garcia-Bernardo J., Heemskerk E. (2020). Does it pay to be a multinational? a large-sample, cross-national replication assessing the multinationality–performance relationship. *Strategic Management Journal*.

[64] Cheung Y.-L., Kong D., Tan W., Wang W. (2015). Being good when being international in an emerging economy: the case of China. *Journal of Business Ethics*.

[65] Mishra S., Modi S. B. (2013). Positive and negative corporate social responsibility, financial leverage, and idiosyncratic risk. *Journal of Business Ethics*.

[66] Sial M. S., Chunmei Z., Khan T., Nguyen V. K. (2018). Corporate social responsibility, firm performance and the moderating effect of earnings management in Chinese firms. *Asia-Pacific Journal of Business Administration*.

